# RNN Language Processing Model-Driven Spoken Dialogue System Modeling Method

**DOI:** 10.1155/2022/6993515

**Published:** 2022-02-26

**Authors:** Xia Zhu

**Affiliations:** Foreign Language Department, Guangzhou Huashang College, Guangdong 511300, China

## Abstract

Speech recognition and semantic understanding of spoken language are critical components in determining the dialogue system's performance in SDS. In the study of SDS, the improvement of SLU performance is critical. By influencing the factors before and after the input text sequence information, RNN predicts the next text information. The RNN language model's probability score is introduced, and the recognition's intermediate result is rescored. A method of combining cache RNN models to optimize the decoding process and improve the accuracy of word sequence probability calculation of language model on test data is proposed to address the problem of mismatch between test data and training data in recognition. The results of the experiments show that the method proposed in this paper can effectively improve the recognition system's performance on the test set. It has the potential to achieve a higher SLU score. It is useful for future research on spoken dialogue and SLU issues.

## 1. Introduction

Spoken Dialogue System (SDS) is composed of automatic speech recognition, spoken language understanding (SLU), dialogue management, language generation, speech synthesis, and so on. SLU performance is very important for SDS. The SLU system is a key component of SDS, which aims to help the computer “understand” the text recognized by the speech recognition module [1]. An important task in SLU is to automatically extract and classify semantic intentions or to fill in a set of parameters or slots embedded in the semantic framework so as to achieve the goal in man-machine dialogue [2]. Although related researchers have conducted research for many years, the task of slot filling and intention determination in SLU is still a challenging problem. The traditional methods to solve SLU are mainly conditional random fields, hidden Markov models, and other traditional methods based on statistics [3]. Natural language understanding is an important factor that determines the usability and naturalness of human-computer SDS. Its robustness directly affects the success rate of dialogue and the user-friendliness of the system [4]. However, due to the randomness of user sentences in spoken dialogue and the imperfection of speech recognition module, the traditional whole sentence analysis method cannot achieve a correct understanding of user sentences, but it is necessary to introduce a robust understanding mechanism to extract the key information in sentences. With the rise of deep learning, the application of Neural Networks (NN) training in the field of Nature Language Processing (NLP) has achieved great success. People began to explore different functions of NN.

With the rapid development of artificial intelligence, there are countless tasks in our society that need to process serialized data [5].The main goal of the early language calculation method is to automatically analyze the language structure and develop basic technologies like machine translation, speech recognition, and speech synthesis [6]. Researchers can use these technologies to create SDS and speech-to-speech translation engines in practical applications, mine social media content for health or financial data, and identify customers' feelings about products and services [7]. The goal of SLU is to automatically identify the fields, categories, and intentions of users' spoken language in order to express natural language and then extract related concepts in order to achieve the goal of system understanding of users' language. Through speech recognition, the computer converts it into corresponding text information, which is then processed by SLU. In recent years, the NN method has demonstrated remarkable performance in a variety of Natural Language Processing (NLP) tasks, particularly the method based on Recurrent Neural Networks (RNN), such as language model, language semantic understanding, and machine translation [8]. This paper employs RNN and its variants to improve the performance of SLU. On this foundation, an RNN-based SDS language understanding method is proposed.

An important task in SLU is to automatically extract and classify semantic intentions or to fill in a set of parameters or slots embedded in the semantic framework so as to achieve the goal in human-computer dialogue [9]. RNN has great advantages in extracting sequence information of natural language characters and using it to build mathematical models to solve corresponding problems [10, 11]. RNN has been verified to have a remarkable effect in solving the serialization problem. In this paper, an algorithm based on recurrent neural network is proposed, which stacks multiple nodes at one time node to deepen the complexity of nonlinear transformation. This method can store longer-term information with fewer parameters by adding storage history state information. According to more information obtained, feature information is extracted to increase the effectiveness of obtained information, improve the accuracy of SLU, and shorten the experimental time. The feature fusion network structure is applied to the data set for SLU experiment. Experimental results verify the effectiveness and reliability of the algorithm.

## 2. Related Work

A new framework for understanding probability was proposed in the literature [12]. A two-level search and comprehension algorithm is also used by the framework. The concept map is created at the second level using a rule-based tree expansion robust syntactic analysis algorithm in order to effectively obtain the overall structure information of the sentence. It solves the problem of a sentence's meaning being ambiguous and it being difficult to accurately extract the sentence's semantic information. To improve the robustness of language comprehension in SDS. Literature [13] proposed a two-level search understanding algorithm. Concept bundling is used to generate the concept map in the first level, and some interference components on the word map provided by the recognition module are removed. The improved robust syntactic analysis based on tree expansion is used to search for the best understanding result at the second level. The literature [14, 15] primarily investigates and implements the related technology of the SLU system's slot filling task. A joint model based on a two-way long- and short-term memory network and label splitting was proposed in the literature [16]. Furthermore, due to the ATIS data set's low-resource characteristics, an attempt was made to introduce external semantic information using foreign pretraining word vectors. An improved RNN language model based on context word vector features was proposed in the literature [17]. Enhance the RNN model's structure by adding a feature layer to the input layer. In response to the issue of language models' poor adaptability to different corpora, literature [18] proposed an adaptive method based on the CNN language model. Literature [19] proposes an RNN that uses external memory to improve memory ability. Literature [20] proposed a feature fusion-based RNN on the basis of RNN and introduced the application of the structural principle and method in SLU. Literature [21] proposed a feature fusion RNN structure based on the analysis of the basic RNN and its LSTM network and GRU network structure. Literature [22] uses adaptive data to adjust the parameters of the general background model and extracts topic features in the adaptive data to join the adaptive training of the RNN language model, enhances the model's ability to describe the adaptive corpus, and improves the language model's ability to adaptability under the corpus. Experimental results show that this method can improve the system's language recognition effect. Literature [23] mainly introduces the principle and performance index of SLU and the structural principle of basic RNN, mainly introduces two basic RNNs in detail, and analyzes its main methods. Literature [24] successfully trained a language model on a text corpus using feedforward NN. By mapping discrete words into continuous real number vectors, it successfully overcomes the impact of data sparseness on statistical modeling and at the same time solves the dimensionality disaster of model parameters' problem. Literature [25] compares the NN language model with other language models and finds that the NN model is compared with other models. For example, when the cache model or the part-of-speech-based model is combined, the resultant hybrid model has a better effect. The article summarizes the key and related research progress of the SLU task and compares the structure and principle of RNN with different structures. Propose an SDS language understanding algorithm based on RNN. The input is sent to the hidden layer for training to obtain a feature representation; then the feature information is sent to another hidden layer for training along with the source input and historical output information; finally, it is sent to the output layer to get the result. Select the data set and performance evaluation method widely used in this field and compare it with several other advanced models on the data set. The results show that the proposed RNN is effective for SLU tasks and has good accuracy and robustness.

## 3. Methodology

### 3.1. SDS

Oral English is the most direct and simple communication medium for people to communicate with each other in their daily lives. People can get information through language communication, which is one of the most important communication ways [26]. Based on this, whether people can communicate with computers directly is one of the research directions in the field of artificial intelligence, and spoken language is the natural language between people. In oral conversation, the speaker's psychological state inferred from various information can also be used to supplement the system's knowledge about the content of user statements [27].

The purpose of SLU module is to extract semantic information from the user's sentences, that is, to identify the intention of the input sentence and extract the corresponding semantic slot concept. The main function of SLU is to analyze sentences' input by users, extract semantic information, and obtain semantic representation. For the whole SDS, the key parts are SLU and dialogue management part [28]. Research shows that deep learning can extract high-level features from shallow features because of its special hierarchical structure. The problems of lack of information and excessive dimension in semantic representation of unified text have been well developed in the fields of image, pronunciation, and so on. At the same time, it has achieved some research results in the field of NLP and shows more potential application value.

SLU is an important component of the dialogue system, and its purpose is to allow the computer to “understand” the input language as if it were spoken by a human. As a result, SLU's performance is closely linked to that of the dialogue system. SLU research can help people apply SDS more accurately, which is more convenient for people's lives and work [29]. SLU's goal is to automatically identify the fields, categories, and intentions of users' oral natural language expressions and then extract related concepts in order to achieve a systematic understanding of the language they use. Domain detection, intention identification, and slot value filling are the three main components of SLU. Slot filling is a labeling task, while domain detection and intention identification are classification problems. The term “slot filling” refers to the practice of marking every word in a sentence [30]. Different semantic representations are used for different SLU tasks. We can use the semantic framework and semantic slot that conform to the semantic structure of the SLU task to model the input intuitively and clearly in the simple understanding task. This framework and semantic slot approach, on the other hand, are no longer suitable for more complex SLU tasks, such as tasks with long phrases.

The first step in a man-machine dialogue system is SLU. Its primary function is to analyze the user's conversation and collect other relevant data about conversation behavior and tasks. According to the information, the dialogue management part updates the current state of the dialogue and generates a dialogue strategy. The dialogue generation part outputs the natural language generated by the dialogue management strategy to the user. Three parts constitute a complete task-driven man-machine dialogue system, and each part has an important influence on the performance of the whole man-machine dialogue system, as shown in Figure 1 below.

Deep Neural Network (DNN) is a successful SLU model applied in NLP field. The biggest feature of DNN is that it can train massive data and then extract the feature information of these data by learning a lot of data. A remarkable feature of NLP applied deep learning is that the input comes from a large number of lexical symbols, which leads to the initial work of Neural Networks (NN) language modeling; that is, these lexical symbols are distributed through learning in the input or output layer, and these embedding and tasks are jointly trained and learned. Following this principle, various network architectures and training methods have been successfully applied.

The main difference between RNN language model and feedforward NN language model lies in the different representations of the historical information of words. In feedforward NN model, the representation method of historical information is similar to that of *n*-gram model, and the first *n* − 1 words are still used. RNN model, on the other hand, obtains historical information through the constant circulation of hidden layer and learning from it. In RNN, the hidden layer can represent historical information, not just the first *n* − 1 words. This model can theoretically represent longer context information.

RNN is an NN structure composed of an input layer, a circulation layer, and an output layer. Among them, the input layer reads each input word and the probability that the output layer generates the corresponding semantic tag. The most prominent feature of RNN is that the current predicted value can be obtained through the common information of the previously input words and the current input words. From the information processing ability of the network, the nodes in the network include input nodes, which are nodes that connect the outside world with the internal network structure of the network; implicit layer nodes and output nodes are nodes with processing capability. The RNN structure of feature fusion is shown in Figure 2.

SDS is like a communication tool for communication between human beings and machines. Through this communication tool, computers can communicate with human beings without obstacles, and computers can give correct answers to various demands of human beings. SDS will meet different users, and different users will have different speech habits. Moreover, dialogue systems usually have to face a lot of first-time users, and first-time users are generally not familiar with the “capabilities” of dialogue systems.

RNN can theoretically predict current word tags based on arbitrarily long historical data. However, because the weight parameters are updated using the random gradient descent method, there will be issues with gradient disappearance and explosion, resulting in the error information being unable to be transmitted far away in the back propagation. At the same time, it restricts RNN's storage and memory capabilities. The accuracy rate is the ratio of relevant labels to all labels trained by NN, which measures the experiment's accuracy rate; the recall rate is the ratio of trained related labels to all related labels, which measures the experiment's recall rate. To put it another way, the accuracy rate is the number of trained labels that are correct, while the recall rate is the ratio of trained correct labels to all correct labels.

### 3.2. SLU Algorithm Based on RNN

A careful analysis of the sentences of the participants in the oral conversation shows that the variability of sentence structure is mainly caused by two reasons: (1) flexibility of word order and (2) frequent use of nonkey components such as colloquial words, auxiliary words, and parenthesis. The key components in the field often have relatively stable structures. Language understanding system is to process and output the input sentence and predict the tag of each word in the sentence. Generally, the input and output of these tasks are one-to-one correspondence, the input is a sequence of words, and the output is the corresponding tag sequence.

The function of nonlinear NN is more powerful than that of linear NN. The main reason is that nonlinear network can distinguish the nonlinear boundary between different data. With nonlinear NN structure, unlike linear NN, neurons with nonlinear activation function have strong learning ability, which can learn new representations through the nonlinearity of several hidden layers. This is because the input and output of the nonlinear activation function are mapped from one limited range to another.

The number of neurons and activation function in each layer of the NN, as well as between each layer, are mostly determined by the different task types. What kind of function can we use if it is a classification task? There will be different activation functions if it is a regression task. In general, only the best sentences generated by the recognition module are processed, but it is difficult to make use of the word graph's wealth of information. It is decided to use two-level processing. As the understanding result, the word graph is first transformed into a concept graph, and then an optimal path is searched on the concept graph using the concept binary grammar. The purpose of long-term dependence of information can be achieved by putting forward three gate units, the input gate, the forgotten gate, the output gate, and the corresponding cell state, and the gradient problem of RNN can be effectively solved by increasing the state of control unit.

The network structure of the model includes input layer, hidden layer, and output layer. The network does not calculate in the input layer and preprocesses the training corpus according to a certain representation; then, the calculation formula of the output of the input layer is

(1) $$\begin{array}{c} x\left(t\right)=w\left(t\right)+s\left(t-1\right). \end{array}$$

The hidden layer of the RNN processes the information sent by input neurons, and the output layer is used to represent the network's output results. The neurons between layers in the network communicate via synapses, and the layers are linked by a weight matrix. The formula for the hidden layer and the output layer is as follows:

(2) sjt=f∑iwitu+ji∑lslt−1wjl,ykt=g∑isjtvkj.

In which *f*(*z*) is sigmoid activation function *f*(*z*)=1/1+*e*^−*z*^. *g*(*z*) is sigmoid activation function *g*(*z*_*m*_)=*e*^*z*_*m*_^/∑_*k*_*e*^*z*_*m*_^. *i*, *j*, and *k* represent the number of neurons in each layer. The output of the network is expressed in matrix form, and the above formula can be rewritten as

(3) $$\begin{array}{c} s\left(t\right)=f\left(Uw\left(t\right)+Ws\left(t-1\right)\right),\\ y\left(t\right)=g\left(Vs\left(t\right)\right). \end{array}$$

The output vector *y*(*t*) represents the probability distribution *P*(*w*(*t* + 1) of the word to be predicted *w*(*t* + 1) given the current word *w*(*t*) and historical information *s*(*t* − 1))∣*w*(*t*), *s*(*t* − 1). The time complexity of each step during model training and testing is proportional to

(4) $$\begin{array}{c} O=H\times H\times H\times V=H\times \left(H+V\right), \end{array}$$

where *H* is the size of the hidden layer and *V* is the size of the vocabulary.

At the first level, based on the word map given by the recognition module, the concept is bound according to the concept rules, and all possible concept candidates in the sentence are obtained, and the concept map is generated. In the second level, according to the sentence-level rule set, a robust syntax analysis algorithm based on tree expansion that can skip noncritical components is used to search for the optimal whole sentence comprehension result on the generated concept map. In RNN structure, the state of information is mainly nonlinear activation of input information. Except for nonlinear property, the state of information can only be updated through external input. Therefore, the storage state is added in the loop layer to store and update the historical information. While adding external information input sources, different nonlinear processing information flows are added so that long-term context storage information can be obtained. Long-term historical information can be stored and new information can be added through the added information flow. The current input information and the stored historical information are processed nonlinearly together, and more feature information that can express the input concept can be obtained through the processing and activation of nonlinear functions.

When the understanding module receives a new word graph, it first creates an empty concept graph; then, it uses the bottom-up chart syntax analysis method to analyze all of the arcs in the word graph according to the defined concept rule set and merges several word arcs that can be combined into a single concept into a concept arc. By weighting the input data, the perceptron activates the output vector, which contains information about the input data. The score is calculated and added to the concept map's corresponding nodes. The interaction between the unit that stores long-term historical information and the loop node can provide the most effective feature information.

The ability of a model trained on a given data set to run on previously unseen data that is similar to the training data is referred to as generalization. The following factors affect NN's generalization ability in order to make it more applicable: (1) NN's structural complexity, capacity, and scale. (2) Sample quality, NN's information content is the sum of all samples trained in the network. The stronger the generalization ability of NN, the more information content in the training samples. (3) The starting weight. (4) Hours of study time, the time it takes for a NN to learn is another factor that influences the network model's ability to generalize.

The learning part consists of the following adjustment parameters of RNN with *n* output layers.

(5) $$\begin{array}{c} \Theta =\left\{E,h^{\left(1\right)}\left(0\right),U^{\left(1\right)},U^{'\left(1\right)},\ldots ,h^{\left(H\right)}\left(0\right),U^{\left(H\right)},U^{\prime }\left(H\right),V\right\}. \end{array}$$

To be precise, the shape of the matrix is (4) and (5).

(6) $$\begin{array}{c} U^{\left(1\right)}\in M_{d_{h}\times d_{e}\left(2d+1\right)}\left(R\right)U^{'\left(1\right)},\ldots ,U^{\left(H\right)},U^{'\left(H\right)}\in M_{d_{h}\times d_{h}}\left(R\right), \end{array}$$

(7) $$\begin{array}{c} V\in M_{N\times d_{h}}\left(R\right). \end{array}$$

For training, use random gradient descent. After calculating the gradient for each sentence in training set *D*, update the parameters to minimize the negative log likelihood. A sentence is considered as a word tuple and a slot tuple.

(8) $$\begin{array}{c} L\left(\Theta \right)=-\sum_{\left(S,W\right)\in D}\sum_{t=1}^{T}\log\;P_{\Theta }\left(s_{t}|l_{0}^{t+d}\right). \end{array}$$

The length of each sentence may vary from one training sample to another, and the window size of context words is a superparameter.

Because the concept extraction and sentence comprehension are handled hierarchically, only 300 rules are used at the sentence level, which basically covers all kinds of user input situations in this field. After obtaining the concept map of the current user sentence, we do not simply search for an optimal path on the concept map according to the concept binary grammar as the final understanding result, but search the sentence space composed of the concept map by introducing sentence-level rules and adopting the improved robust syntax analysis method based on tree expansion. The information about context is mainly obtained by processing the input information and the saved context state together to obtain the feature information of context. These historical feature information are activated by nonlinear functions, and finally more detailed and specific feature information is obtained. Finally, the training results of the hidden layer are sent to the output layer for judgment and calculation.

The effect of network training can be influenced by data preprocessing in some cases. As a result, some data preprocessing decisions must be made. However, network training after preprocessing can sometimes achieve the same effect as training and learning the data directly, and data without preprocessing can sometimes achieve better results, making preprocessing redundant. In an RNN structure, the unit structure with the function of saving historical information primarily sends the current moment's input data and the previous moment's historical storage data to the storage unit for activation processing. The activation function is a nonlinear function in this case, and activation of the activation function yields feature information that has a strong correlation with the input historical data and current data.

## 4. Results Analysis and Discussion

In SDS, the meaning of the user's current statement has a strong correlation with the conversation history, so this information can be used to infer the meaning of the current statement. In order to bind concepts, which are the key components in the word map, we first need to define a group of concepts in current application fields and their corresponding composition rules. In order to prove the practicability of the RNN model proposed in this paper, this paper uses the data set widely used in experiments such as SLU, that is, the experiment of oral semantic understanding on the data set of Air Travel Information System (ATIS).

Check the analysis results of concept map. If there is a whole sentence analysis result, select the path with the highest score for semantic extraction; otherwise, search for an optimal path on the concept map and perform semantic extraction according to the context of dialogue management. The tuning parameters in the experiment include the number of units in the hidden layer. In this experiment, the number of units in the hidden layer is set to 200, the dimension of the word vector in the word embedding layer is set to 200, and the back calculation steps of the back propagation algorithm applied in this paper are set to 10. The weight matrix and offset of NN are updated by back propagation, respectively. In this section, the traditional Condition Random Fields (CRF) is compared with Convolution Neural Networks (CNN) and this model. In order to observe the process of network training and learning more intuitively, the performance index of the network is described by describing the change process of F1 value, and the line chart is drawn as shown in Figure 3.

Considering the guiding role of historical information in SDS and the structural characteristics of user sentences in the field of train information query, it is decided to use two aspects of information to bias the search space: user intention inference based on dialogue history and sentence feature phrases. At the same time, the relationship between entropy of training sets and iteration times of different models is compared to compare their convergence speed. The results are shown in Figure 4.

The training set entropy is expressed in logarithmic form. Compared with other models, the proposed model has lower training entropy and the best convergence speed. Experimental results show that this model has good accuracy and robustness and is suitable for SLU tasks. Defining the dialogue state based on the recent dialogue history greatly reduces the dimension of the state space, but it only uses limited local historical information, which reduces the accuracy of prediction. In order to give an efficient and accurate prediction of subrule set by using historical information as much as possible, a new prediction idea is proposed, which is not based on each specific historical state of conversation but based on the preconstructed user plan model to infer the user's intention.

CRF is the most commonly used method to deal with sequence tagging, and it has achieved good results in sequence processing. In this paper, CRF model, RNN, and CNN are used to perform feature fusion experiments on ATIS dataset. By changing the neurons in the network structure to process the data, the experimental results are shown in Figure 5.

The results of the above experiments show that the deep RNN feature fusion model outperforms CRF and CNN in SLU. When the optimal path analysis results are unavailable, this algorithm analyzes all concept maps, which saves time by not having to search all sentence spaces contained in concept maps. The pruning-while-expanding strategy can greatly reduce the scope of the search space during the analysis process. The precision, recall, and *F*1 performance indexes used in this experiment to assess oral semantic understanding are precision, recall, and *F*1. The proportion of correctly marked words to all correctly marked words is referred to as the accuracy rate, while the proportion of correctly marked words to all correctly marked words is referred to as the recall rate. In the labeling of evaluation data, the recall rate is the proportion of correct labels. The following is how *F*1 is written:

(9) $$\begin{array}{c} F_{1}=\frac{\mathrm{2\times precision\times recall}}{\mathrm{precision+recall}}. \end{array}$$

In the process of dialogue, every time the user inputs a new sentence, the system reinfers and updates the user's intention according to the understanding result of the sentence and the historical information of the user's intention and then predicts the possible input of the next sentence by the user according to the inferred user's intention to determine the corresponding subrule set. Because the user's intention inference information and sentence feature phrase information based on dialogue history come from two independent information sources, the two kinds of information can be directly combined to restrict the search space. The three models are compared.  Figure 6 shows the comparison of the accuracy of different models.  Figure 7 shows the comparison of recall rates of different models.  Figure 8 shows the *F*1 comparison of different models.

The SLU experiment on ATIS data set can be seen from the above results. The experimental results obtained by RNN model in this paper are always better than those obtained by CRF and CNN methods. The superiority of this method is verified. In this chapter, we propose the DNN structure of feature fusion through the NN structure described earlier and combine the features of DNN to concentrate multiple features in a time node for calculation. This paper introduces the experiments of RNN, CNN, and CRF network structures on the database. The results show that the proposed RNN with external memory is effective for SLU tasks, has good accuracy and robustness, and has certain advantages in training error and convergence speed.

## 5. Conclusions

The basis of SLU is to represent words as symbols that can be read by machines, that is, the representation of words. In the task of SLU, it is mainly to label each word in the input text sentence with a corresponding label, and the most effective model algorithm to solve SLU is RNN. On this basis, this paper proposes an RNN that can store long-term historical information. The NN structure can solve the problem of gradient disappearance with fewer parameters. Based on the unified statistical framework of search, the information of user's intention inference and sentence feature phrases are introduced to constrain the search space, which further improves the robustness and real-time rate of understanding. At the same time, it achieves better results than CNN and GRU. In order to further improve the robustness and real-time rate of understanding, the information of user intention inference based on dialogue history and sentence feature phrases are introduced in the second level to restrict the scope of search space. The path is evaluated and pruned based on the statistical framework, which can ensure the real-time performance of the algorithm and obtain high understanding accuracy. The model in this paper is compared with other models on ATIS data set. Experimental results show that the SLU method based on RNN proposed in this paper is effective for SLU tasks and improves the robustness and accuracy of the original model. And the *F*1 value is significantly improved. The next task of this paper is to apply RNN to other NLP tasks in order to increase the universality of RNN network structure.

## Figures and Tables

**Figure 1:** Man-machine dialogue system.

**Figure 2:** RNN structure of feature fusion.

**Figure 3:** Comparison of training results of three models.

**Figure 4:** Comparison results of different models.

**Figure 5:** Model depth feature fusion.

**Figure 6:** Accuracy comparison of different models.

**Figure 7:** Comparison of recall rates of different models.

**Figure 8:** *F*1 comparison of different models.

## Data Availability

The data used to support the findings of this study are included within the article.
